# Performance Analysis of Ovarian Cancer Detection and Classification for Microarray Gene Data

**DOI:** 10.1155/2022/6750457

**Published:** 2022-07-15

**Authors:** M. Kalaiyarasi, Harikumar Rajaguru

**Affiliations:** Bannari Amman Institute of Technology, India

## Abstract

The most common gynecologic cancer, behind cervical and uterine, is ovarian cancer. Ovarian cancer is a severe concern for women. Abnormal cells form and spread throughout the body. Ovarian cancer microarray data can diagnose and prognosis. Typically, ovarian cancer microarray data contains tens of thousands of genes. In order to reduce computational complexity, selecting the most critical genes or attributes in the entire dataset is necessary. Because microarray datasets have limited samples and many characteristics, classifier detection lags. So, dimensionality reduction measures are essential to protect disease classification genes. In this research, initially the ANOVA method is used for gene selection and then two clustering-based and three transform-based feature extraction methods, namely, Fuzzy C Means, Softmax Discriminant Algorithm (SDA), Hilbert Transform, Fast Fourier Transform (FFT), and Discrete Cosine Transform (DCT), respectively, are used to select relevant genes further. Six classifiers further classify the features as normal and abnormal. The NLR classifier gives the highest accuracy for SDA features at 92%, and KNN gives the lowest accuracy of 55% for SDA, Hilbert, and DCT features. With correlation distance feature selection, the NLR classifier attains the lowest accuracy of 53%, and the highest accuracy of 88% is obtained by the GMM classifier.

## 1. Introduction

Cancer is the world's top public health risk. The causes of cancer are unknown. Hence, there is no efficient way to diagnose it. As a result, early cancer diagnosis improves the chances of full recovery and survival rate. Therefore, early cancer diagnosis is critical to increasing the survival rate [1]. According to Shabir S, Gill PK et al., in 2012, it was diagnosed that there were 239,000 cases of ovarian cancer worldwide, with 600,000 women living within five years of a diagnosis. By 2035, ovarian cancer is expected to rise to 55% and 67% of fatalities [2]. Ovarian cancer will rise to pandemic proportions and universally become a problem. Between 2012 and 2030, the number of new cancer cases is expected to rise by 70%, from 14 million to over 22 million, putting an ever-increasing burden on low- and middle-income countries.

Women's cancers account for 2.5 percent of all cancers. Women are getting cancer at a higher rate than ever before, measured as a percentage of the population. Ovarian cancer ranks fifth, while breast cancer ranks eleventh among cancer-related severe cases in women [3]. African American women have slightly higher mortality rates than Caucasian women. A pelvic exam, imaging tests such as transvaginal ultrasound, CT, PET, MRI, microscopic examination of a tissue sample, CA-125 blood test for tumour markers, blood test for gene changes, and gene expression analysis are used to diagnose ovarian cancer [4].

Microarrays are found to be better at detecting and classifying cancer than other image processing tools. Thus, microarray data is used in this study. Gene expression analysis is one example of a large-scale experiment that looks at a lot of genes at the same time. DNA microarrays are widely used in biological and medical research to examine gene expression in cells and diagnose disorders such as cancer. In functional genomics, enormous amounts of data from numerous biological investigations are analyzed. Microarray technology uses hybridization to monitor hundreds of genes on a tiny chip. Gene expression microarrays have a lot of potential to help doctors make decisions about cancer diagnosis and treatment [5]. An aberrant tissue is one that has gene expression alterations because of the fluctuation of gene expression. Each cell's protein components determine its function and response to external stimuli. The genes expressed by an organism's cells determine its behaviour [6]. Gene expression can be quantified using nucleic acid microarrays that track DNA or RNA quantities in distinct cells over time. Microarray experiments include systematic causes of variance that should be addressed before any study is done. The workflow of an experiment on microarrays involves, in addition to the measuring technique, an intensive data analysis step. The microarray targets hybridization with subsequences (probes) of genes in the entire genome on a microarray blade, with each gene having its own fluorescent spot. A microarray image called a probe, combined with a fluorescent tag, is generally compared to a reference image, recorded with the second fluorescent tag, in a two-colour microarray experiment. The intensity of fluorescent light is used to determine gene expression levels using specific microarray image processing techniques [7]. The extraction of point intensity characteristics and data normalization are for estimating gene expression levels and determining pixels belonging to the microarray spot or its nearby backdrop. After normalization, each row in the preprocessed data indicates a gene expression value at distinct time points or experimental conditions. Many studies have 4000–8000 gene rows and 4–80 gene expression values [8].

The primary objective of this research is to devise a system that can correctly categorize various forms of cancer. The data relating to cancer should be organized in such a way as to make it less difficult for patients to obtain treatment and to reduce the associated risks. If the data from the microarray includes genes that are not relevant or that have a lot of noise, the accuracy of the classifier will be reduced as a result. Therefore, efficient methods of gene selection and feature extraction will be able to guide you in selecting characteristics that are useful. Additionally, in order to acquire a perfect classification of the data pertaining to cancer, it is necessary to make use of various procedures and investigate whether or not they offer improved classification accuracy. The results of this work provide the best performance in terms of the accuracy of classification.

This research study uses two clustering-based and three transform-based feature extraction methods in order to be able to select an informative gene subset while eliminating/declining redundant or irrelevant genes and to be able to improve the performance of microarray high-dimension data classification. Six classifiers further classify the features as normal and abnormal.

To exploit the benefits of this technology, researchers are developing and employing more precise decision support models. It has been used to predict ovarian cancer. This research highlights the need for a computer-aided approach for ovarian cancer classification from microarray gene expression. This augments medical professionals and clinical professionals in a speedy diagnostic process.

## 2. Review of Ovarian Cancer Literatures

The following section discusses the most significant studies in the area of ovarian cancer classification. The review of ovarian cancer literature for the last two decades is discussed in this section. According to B.C. Lee et al., for the differentially expressed genes, the microarray analysis in female ovarian cancer provides information on the disease. [9]. H.S. Chon and J.M. Lancaster talked about gene expression studies in 2011 that used microarrays to look for biomarkers for early ovarian cancer [10]. Zhang et al. give an outline of various types of biomarkers that can be used to diagnose ovarian cancer in women [11]. Lee [12] developed a hybrid process of GA, PSO, SVM, and ANOVA to select gene markers and an integrated method by using Fuzzy, LDA, FCM, and *K* Means for gene selection and classification of ovarian types as ovarian tumours (OVT), five ovarian cancers at stage I (OVCAI), and five ovarian cancers at stage III (OVCAIII). Jeng et al. used intelligent algorithms to examine microarray data by Support Vector Regression (SVR) in order to classify stages of ovarian cancer [13]. Tan et al. developed neural networks based on complementary learning (FALCON-AART) for the diagnosis of ovarian cancer, obtaining an accuracy of 91.10% and attaining 78.90% accuracy by blood test [14]. Chuang et al. [15] performed a dimension reduction by Support Vector Regression (SVR) on the ovarian cancer microarray data in order to reduce it from 9600 genes to about 300 genes. Huang et al. [16] performed a machine learning-based microarray analysis of ovarian cancer to identify genetic markers associated with the stages of ovarian cancer. Zhu and Yu used gene patterns to classify epithelial ovarian cancer with the attainment of UBE2I. The mean RQ values were 5.76 and 3.85 [17]. Yu and Chen [18] applied a Bayesian neural network approach to the diagnosis of ovarian cancer using high-resolution mass spectrometry data in order to identify the malignancy, and BNN achieved average levels of sensitivity and specificity of 98.56% and 98.42%, respectively. Vlahou et al. [19] did research to diagnose ovarian cancer by using a classification and regression decision tree categorization of group spectral information to classify the tumour and obtained an accuracy of 81.5% in the cross-validation analysis and 80% in a blinded set of samples. When Deep Convolutional Neural Networks (DCNN) were used to classify the various forms of ovarian cancer from cytological pictures by design, the accuracy of classification models improved from 72.76 to 78.20%, which was done by Wu et al. [20]. Mas et al. conducted a study in which they examined machine learning algorithms *K*-Nearest Neighbors (KNN), Linear Discriminant (LD), Support Vector Machine (SVM), and Extreme Learning Machine (ELM) involving the Fourier Transforms for the categorization of ovarian cancers, giving an accuracy of 58.29%, 85.56%, 87.70%, and 87.70% [21]. Nuhic et al. did research on several categorization strategies for the detection of ovarian cancer, and they did a comparison and found that logistic model trees had the best accuracy at 96.78% [22]. An investigation was carried out by Zhang et al. into the use of ANN in the early diagnosis of ovarian cancer with a sensitivity of 88.9% [23]. Antal et al. [24] investigated the potential and limitations of using Bayesian networks for the diagnosis of ovarian cancer in a clinical setting and attained 95.2% in Receiver Operator Characteristics (ROC). Osmanovic et al. used decision tree (DT) classifiers to diagnose ovarian cancer in individuals who had previously undergone surgery. They used historical data to make their determination and gave the accuracy as 77.2% for both the J48 and the LMT classifier [25]. Thakur et al. were able to detect ovarian cancer early because of the use of feed-forward artificial neural networks with an accuracy of 98% [26]. Kusy [27] applied the SVM to the categorization of ovarian cancers and published his findings. According to Nabawy et al. [28], the epithelial ovarian cancer stage subtype classification was achieved through the use of gene expression analysis and boosting algorithms, which outperforms the other types of classifiers with an accuracy of 80%. Park et al. [29] developed an intraoperative diagnosis assistance tool for ovarian cancer based on microarray data, in which they used a multicategory machine learning algorithm in which the SVM model had the best accuracy of 97.3%.

Arfiani and Rustam [30] developed a classification system for ovarian cancer that included a bagging method with 100% accuracy for 90% of the training data and a random forest that reached 98.2% accuracy for 90% of the training data. Acharya et al. [31] developed a novel online paradigm for ovarian tumour characterization and classification using ultrasonography with a DT classifier that presented a high accuracy of 97%. Cohen et al. [32] investigated the use of 3D power Doppler ultrasonography to improve the accuracy of diagnostics for ovarian cancer. As per Renz et al., ovarian disease can be grouped by a Multi-Layer Perceptron (MLP) classifier and attain a 92.9% accuracy. [33]. Assareh and Moradi [34] have developed a method for extracting the most effective fuzzy if then rules from mass spectra of blood samples for the purpose of early detection of ovarian cancer. The classifiers used for these blood samples are KNN and LDA with 100% accuracy. When Meng et al. [35] looked at the features from ovarian cancer proteome mass spectra, they found that 98% of the time, they were able to detect the disease. They also found that 95% of the time, they were able to identify the disease. Kim et al. [36] investigated the use of Logistic Regression to combine various biomarkers for the early identification of cancer at an early stage in order to improve early detection rates. The LDA classifier has a 78.38 percent accuracy rate.

RabiaMusheer Aziz has done the classification for different cancer data with ABC and ICA with cuckoo and found the 93.67% as high accuracy [37]. Yan Ma et al. developed a method to identify the ovarian cancer by noninvasive serological diagnostic approach using TAA antigens [38]. According to Rabia Aziz et al., ICA + ABC is used for gene selection and classification with ANN classifier [39]. Douglas V. N. P. Oliveira investigated the gene profile using the biomarkers [40]. RabiaMusheer Aziz et al. have done the classification Independent Component Analysis (ICA) and Artificial Bee Colony (ABC) with the maximum accuracy of 97.12% (20 genes) of ABC and 95.11% (28 genes) of ICA [41]. Md Shahjaman et al. investigated for ovarian cancer to identify the improved core biomarkers [42]. RabiaMusheer Aziz investigated on nature-inspired algorithm and developed cuckoo search algorithm [43]. Deng, Xiongshi et al. developed the hybrid gene selection approach using XGBoost and multiobjective genetic algorithm for cancer classification [44]. Alhenawi, Esra'A. et al. have done a review on feature selection and classification of microarray gene data for cancer [45]. Prabhakar, S. K. and Lee, S. W. have done the investigation on optimization algorithms for gene data extraction and classification [46].

There are various algorithms for gene selection and cancer classification that make use of a microarray that can be found in the research literature. Many computer methods have been developed for gene selection, although most focus on data samples while ignoring gene correlation. The correlation distance is calculated after the gene selection. Finally, the classification algorithms Gaussian Mixture Modelling, Detrended Fluctuation Analysis, Nonlinear Regression, Bayesian Linear Discriminant, Logistic Regression, and *K*-Nearest Neighbor (KNN) were able to improve the performance of microarray high-dimension data classification. The performance matrix of six classifiers gives the better analysis of accuracy.

In Section 3, materials and the method are discussed. Feature extraction by clustering- and transform-based techniques for further gene selection is presented in Section 4. Classification techniques are analyzed in Section 5. Results and discussions are given in Section 6.

## 3. Materials and Methods

### 3.1. Methodology

Microarray datasets include a wealth of genomic information that, if correctly evaluated, could revolutionize science and healthcare. Microarray tests have been performed in order to better understand the genetic causes of cancer and to categorize cancerous and noncancerous cells in order to better treat cancer patients. Over the last decade, machine learning algorithms for microarray data analysis have been actively investigated. Various methods have been investigated to (i) discriminate among malignant and noncancerous samples and (ii) classify cancers into groups.

Prominent genes are selected by the ANOVA method for microarray gene data. The features are extracted from the selected genes by two clustering-based feature extractions, Fuzzy C Means and Softmax Discriminant algorithm, and three transform-based feature extraction techniques, Hilbert, Discrete Cosine Transform, and Fast Fourier Transform. By finding the correlation distance, feature selection is possible. Based on the extracted features, the genes are classified with and without feature selection. To get better accuracy and to solve nonlinearity problems, linear algorithms are used in this work for the classification of microarray gene data. The performance metrics from the classifiers are analyzed.  Figure 1 depicts a schematic representation of the classification methodology for ovarian and normal tissues based on microarray gene data.

The proposed method in this research, MATLAB 2017b, is used in experiments on preprocessing the datasets. This tool is used to find features and classify them. A desktop computer with 64-bit Windows 10 and an Intel (R) Core (TM) i5-Intel(R) Core(TM) i3-3220 CPU @ 3.30 GHz and 8 GB of RAM was used for the tests.

### 3.2. Database of Ovarian Cancer

A few genomic datasets are freely accessible from the National Center for Biotechnology Information (NCBI), Stanford University, and the European Bioinformatics Institute (EBI). For the purposes of this investigation, a microarray ovarian cancer dataset was used. The microarray ovarian cancer database is accessible in ovarian cancer sample microarray gene data E-GEOD–69207, which was collected by the European Bioinformatics Institute (EMBL-EBI) and is openly accessible [47, 48]. This is an International Governmental Organization (IGO) which gives the entire molecular database freely. Array express was used to analyze frozen archival epithelial ovarian cancer data. A total of 100 samples, of which 50 samples are normal and 50 samples are ovarian cancer, were obtained, and the genomic data was analyzed using microarrays. To make sure that each sample has the same amount of RNA, the samples are hybridized with materials from an Affymetrix kit.

### 3.3. Gene Selection

Prominent genes are selected by volcano plots for the microarray gene data [49]. These plots help to visualize the outcomes of RNA sequence and additional omics investigations. This volcano plot is a form of scatter plot that illustrates the relationship between *P* value and fold change. *P* value represents statistical significance, and fold change represents the magnitude of the change [49].

Figure 2 shows the volcano plot of ovarian and normal microarray gene data. On the left, genes that are most likely to be downregulated are found. On the right, genes that are more likely to be upregulated are found, and on top of the figure are the most statistically significant genes. After the ANOVA method, out of 33,000 genes, 16,000 genes per sample for normal and ovarian prominent genes were selected.

The next section discusses feature extraction for microarray cancer data. Prior knowledge can be used with feature extraction or feature selection methods to improve the accuracy and complexity of algorithms in cancer data.

## 4. Clustering- and Transform-Based Feature Extraction

Gene expression datasets that are not linearly separated can be solved by choosing the right linear algorithms for better classification. By employing extraction of features, which is a dimensionality reduction technique, it is able to represent key parts of the preprocessed data in the compact form of feature vectors.

The two clustering-based and three transform-based feature extraction methods, namely, Fuzzy C Means, Softmax Discriminant Algorithm (SDA), Hilbert Transform, Fast Fourier Transform (FFT), and Discrete Cosine Transform (DCT), are separately used to select relevant genes further to get the reduced features. The microarray gene data inhibit ambiguity, imprecision, and noise. As a result, using clustering techniques is an important first step in data analysis to reveal natural structures and patterns using Fuzzy C Means and Softmax Discriminant Algorithm (SDA) [50–52].

Dimensionality reduction is promising since it extracts significant data features and reduces processing complexity. For microarray data, the Hilbert Transform, Fast Fourier Transform (FFT), and Discrete Cosine Transform (DCT) are used extensively in voice and image processing for decorrelation, ordering, and dimensionality reduction. Even though the DCT, FFT, and Hilbert Transform algorithms are well-known, their use in identifying microarray ovarian data is innovative. The performance of the above transform methods was analyzed in this research.

### 4.1. Clustering-Based Feature Extraction

Clustering was employed in this work to overcome the redundancy of selected genes. Clustering is the process of grouping entities of low interclass resemblance. A cluster attribute is used to group the attributes so that they are similar in comparison to those of other clusters before applying ranking approaches directly to the attributes of datasets (genes). Although diverse criteria provide varied results in clustering, they all try to group genes based on similarities. Similarity-based clustering is achievable by *K* Means, Fuzzy C Means, C Means, and Possibilistic C Means.

#### 4.1.1. Fuzzy C Means

This FCM algorithm correlates each variable with each cluster by means of a member feature describing the varying strength of the relationship between the various variables and the clusters. As a result, instead of just exclusive partitions, sets of nonexclusive clusters are formed, allowing genes to belong to multiple clusters. It operates by allocating a collection of genes to a given number of clusters, with each gene having the possibility of belonging to more than one cluster, with varying degrees of membership. During this procedure, the algorithm strives to reduce the goal function to its smallest possible value [53]. The goal is to reduce the objective function specified as follows:

(1) $$\begin{array}{c} \overset{p}{\underset{n=1}{\sum }}\underset{k_{m}\in F_{n}}{\sum }x_{mn}^{y}{\left(k_{m}-\mu_{n}\right)}^{2}, \end{array}$$

where *x*_*mn*_ is the degree to which an observation *k*_*m*_ belongs to a cluster *F*_*n*_, *μ*_*n*_ is cluster center, and *y* is fuzzifier.

By the FCM method, 16,000 microarray gene data per sample is reduced to 660 per sample for normal and ovarian for further classification. When FCM clustering is used, the results are significantly improved.

Figure 3 depicts the histogram plot for normal and ovarian cancer data of the FCM feature. From this figure, discontinuity of data is visible. This nonlinearity plot created the necessity to identify the nonlinear classifier to classify the normal and ovarian cancer.

Figure 4 depicts the scatter plot for the FCM feature output of the normal and ovarian cancer data. A scatter plot is to check the clustered nature of data. From this figure, nonlinearity and overlapping of data are depicted. Hence, it is necessary to identify the nonlinear classifier for the classification of normal and cancer data.

#### 4.1.2. Softmax Discriminant Algorithm (SDA)

SDA is the most feasible and effective classifier. The SDA goal is to identify a subset to which a specific test must be applied [54], which is accomplished through classification. Specifically, it is accomplished by comparing and evaluating the distance between the training sample and the test sample. The assignment of the label information is done with the help of a nonlinear transformation of the distance.

Consider the dataset from *s* distinct classes is given by

(2) $$\begin{array}{c} Y=\left[Y_{1},Y_{2},Y_{3},\cdots \cdots Y_{s}\right]\in K^{ab}. \end{array}$$

From *S*^th^ class, the *b*_*s*_ samples are represented by

(3) $$\begin{array}{c} Y_{s}=\left[Y_{1}^{s},Y_{2}^{s},Y_{3}^{s},\cdots .,Y_{b_{s}}^{s}\right]\in K^{ab_{s}}, \end{array}$$

where

(4) $$\begin{array}{c} \overset{s}{\underset{j=1}{\sum }}b_{j}=b. \end{array}$$

Now SDA is defined as

(5) $$\begin{array}{c} h\left(y\right)=\arg\underset{j}{\max}d_{y}^{j}, \end{array}$$

where

*d*_*y*_^*j*^, *h*(*y*) denotes the distance between the testing sample and *j*^th^ class, the identification of *y*, respectively.

(6) $$\begin{array}{c} \left(H\left(y\right)\right)=\arg\underset{j}{\max}\log\overset{b_{j}}{\underset{i=1}{\sum }}\exp\left(-ƛ{\left\|y-y_{i}^{j}\right\|}_{2}\right). \end{array}$$

The objective of SDA is achieved by increasing the nonlinear transformation value of the distance between the testing sample and the *s*-class samples. By the SDA method, the microarray gene data of 16,000 is reduced to 3,300 gene data for further classification.  Figure 5 is the normal probability plot to identify the normal distribution of SDA feature data for ovarian cancer. From Figure 5, the data is left skewed and outliers are identified. So, it is important to make sure the data is the best it can be to get the best classification accuracy.

### 4.2. Transform-Based Feature Extraction

Transform-based approaches are a significant subset of feature extraction techniques that should not be overlooked. In the classification stage, these methods enable the extraction of effective features by removing irrelevant characteristics (transform coefficients). This allows the generalization performance to stay the same while the computational cost goes down [55]. It is possible to separate transform-based methods for feature extraction into linear, nonlinear, supervised, and unsupervised, as well as signal-dependent and independent methods. In this work, Hilbert, Discrete Cosine Transform, and Fast Fourier Transform methods are used for transform-based feature extraction.

#### 4.2.1. Hilbert Transform

The Hilbert Transform (HT) is used as a standard procedure in signal processing. The HT is used to get the analytical representation of the signal and to get the spectrum of the signal without change in the domain. The Hilbert Transform of any signal is not an equivalent representation of the signal; rather, it is an entirely different signal [56]. It is a linear operator that uses the convolution function 1/*πt* to get the real value signal. The Hilbert transform is a ±900 phase shifter for all moving components of the signals without changing their amplitude.

(7) $$\begin{array}{c} H\;\left[a\left(t\right)\right]=a\left(t\right)*\frac{1}{\pi t}. \end{array}$$

*a*(*t*) is a signal, then Hilbert Transform of *a*(*t*) is represented as a *H* *a*(*t*) and it is a convolution of *a*(*t*) with the signal 1/*πt*.

(8) $$\begin{array}{c} H\left[a\left(t\right)\right]=\frac{1}{\pi }\int_{-\infty }^{\infty }\frac{a\left(\tau \right)}{t-\tau }\;d\tau ,\\ H\left[a\left(t\right)\right]=\;\frac{1}{\pi }\int_{-\infty }^{\infty }\frac{a\left(t-\tau \right)}{\tau }\;d\tau . \end{array}$$

This definition says that the transform changes the sign only and does not change our basic results. Also, it finds the imaginary value of a function to have a real value and vice versa. Using the Hilbert method, 16,000 microarray gene data was reduced to 3,300 per sample for further classification.

#### 4.2.2. Discrete Cosine Transform

The DCT method is an approximation of the Kernighan-Lin method to reduce the dimensions. It removes the most significant features of the input and enables a reduction in the complexity of further analysis. This method helps to orthogonalize and minimizes the complexity of a given vector and its components. With the help of the DCT method, the features are extracted by selection of coefficients. It is the most critical and significant step, and it has a significant impact on computation efficiency [57, 58]. DCT is expressed as,for

(9) $$\begin{array}{c} K\left(x\right)=\propto \left(x\right)\overset{S-1}{\underset{u=0}{\sum }}a\left(u\right)\cos\left[\frac{\pi \left(2u+1\right)x}{2S}\right],\\ x=0,1,2,3,\cdots \cdots ,S-1. \end{array}$$

Using the DCT method, 16,000 microarray gene data was reduced to 3,300 per sample for further classification.

#### 4.2.3. Fast Fourier Transform

The best and most popular method for calculating the DFT is the FFT, which can be used in a variety of applications. Time series data can be transformed into the frequency domain by FFT. This approach is useful on many occasions, but utilizing the formula explicitly is inefficient. So this transform evaluates DFT quickly. It divides the DFT matrices into zero factors. As an outcome, it simplifies the discrete Fourier Transform. It is substantially more precise than the discrete Fourier Transform [59]. The FFT equation is

(10) $$\begin{array}{c} x\left(a\right)=\overset{\left(\frac{K}{2}-1\right)}{\underset{i=0}{\sum }}\left[x\left(i\right)+{\left(-1\right)}^{a}x\left(i+\frac{K}{2}\right)\right]Y_{K}^{ai}, \end{array}$$

where

(11) $$\begin{array}{c} Y_{K}^{ai}=e^{j2\pi /K}, \end{array}$$

*K*= FFT points.

The Fourier Transform of the *X*(*f*), time-domain signal *x*(*t*), is given by

(12) $$\begin{array}{c} X\left(f\right)=F\left\{x\left(t\right)\right\}=\int_{-\infty }^{\infty }x\left(t\right)e^{-j2\pi ft}dt. \end{array}$$

The FFT method reduces the 16,000 microarray gene data to 3,300 per sample for further classification.

### 4.3. Statistical Parameters from Feature Extraction

Dimensionality reduction through feature extraction is a type of dimensionality reduction that is used in a specific application. In feature extraction, the primary goal is to extract relevant or significant information from real-world data and present that information in a lower-dimensional space than the original data.

The most accurate and advanced method to predict the cancer for the extracted features is to calculate the statistical parameters. The list of statistical parameters of the clustering- and transform-based feature extraction methods involved is mean, standard deviation, variance skewness, kurtosis, Pearson's coefficient, *t*-test, and sample entropy.

The statistical parameters of cancer data after clustering- and transform-based feature extraction are shown in Table 1. The standard deviation is the gap between categories that are positive and those that are negative. From Table 1, it is observed that the Pearson coefficient is 1 for FFT and DCT in both cases. It shows that they are highly correlated within the classes. It is observed that the nonlinearity comes from the skewness and kurtosis. Sample entropy is a measure of the amount of uncertainty in data. The presence of non-Gaussian is observed from the sample entropy in Table 1. The FFT and DCT give high values of skewness and kurtosis.

## 5. Feature Selection by Correlation Distance

Feature selection reduces the number of input variables in a predictive model. Adding extraneous characteristics reduces the model's accuracy rate, complexity, generalization ability, and generalization capability, and makes the model biased. Choosing features is thus an important stage in developing a machine learning model. Its aim is to find the optimal features for a machine learning model [60].

In this paper, feature selection is done by correlation distance. To determine the distance between the two random variables having limited variances, such as 1, the correlation distance metric is popularly used. This metric is given as *d* = 1 − *a*, while the correlation between the two variables is *a*. A correlation distance is used to find the linear and nonlinear relationships between the random variables. This correlation distance is measured as

(13) $$\begin{array}{c} d\text{cor}\left(X,Y\right)=\frac{d\mathrm{cov}\left(X,Y\right)}{\left[d\mathrm{var}\left(X\right)d\mathrm{var}\left(Y\right)\right]}, \end{array}$$

where *X* and *Y* are the random variables.

By correlation distance, only 45 prominent genes per sample are selected for classification in all feature extraction methods.

## 6. Classifiers with and without Feature Selection

The classification challenge entails the development of a classifier that accepts as an input vector of gene expression and produces as an output a vector indicating the class label of the input sample vector. The six different classifiers are used for the classification of ovarian cancer data with and without feature selection.

### 6.1. Fitness Function

The proposed method's fitness function depends on the classifier's accuracy. If the current fitness value is greater than the previous one, it advances to the next solution. Otherwise, the prior one is retained. Finally, the best predicted gene set is assigned the fitness solution with the highest value. The fitness function (fit) is defined as follows:

(14) $$\begin{array}{c} \text{Fitness}\left(\text{f}\right)=\text{Accuracy}\left(\text{f}\right) \end{array}$$

where Accuracy (fit) is testing data (f) classifier accuracy.

The main objective of this research is to select relevant attribute and improved classification accuracy. Henceforth, the target selection is used for better classification accuracy. The ovarian data is divided into two categories: normal and cancer. This information can be used to determine the target values.

The target *T*_*C*_ is selected with care, with higher values in the range of 0 to 1 being preferred. The following are the criteria that were used in the selection of *T*_*C*_:

(15) $$\begin{array}{c} \frac{1}{k}\overset{k}{\underset{x=1}{\sum }}\mu_{y}\leq T_{C}. \end{array}$$

All of the characteristics of overall (*k*) ovarian cancer data are normalized, and the mean of the normalized data is given by the symbol *μ*_*x*_ in the function, which may be used to categorize the data.

When applying the condition to normal ovarian cases, the target *T*_*N*_ is chosen with lower values in the range of 0 to 1 when using the target *T*_*N*_:

(16) $$\begin{array}{c} \frac{1}{m}\overset{m}{\underset{y=1}{\sum }}\mu_{y}\leq T_{N}. \end{array}$$

The features of the total (*m*) ovarian normal data are normalized, and the equation that can be used for classification says that *μ*_*y*_ is the mean of the data, which can be used for classification.

The value of *T*_*C*_ should be bigger than the values of *μ*_*x*_ and *μ*_*y*_ that were thought of *T*_*C*_ and *T*_*N*_ must be checked to make sure that the difference between the two is either 0 or more than 0.5.

(17) $$\begin{array}{c} \left\|T_{C}-T_{N}\right\|\geq 0.5. \end{array}$$

In this case, the *T*_*C*_ and *T*_*N*_ values are set to be 0.9 and 0.1.

The fitness value (mean accuracy) required for classifier is computed by training with training data and tested by 10-fold cross-validations. Cross-validation *k* times are used for this study. The dataset with the features is first divided into “*k*” points of the same size. Performance in each step is then assessed using k1 groups. Validations are repeated *k* times, with *k* =10 in this case. As a consequence, 90 percent of the data was used for training and 10 percent for testing. Averaging occurs when all performance measures are calculated at the end of the 10-fold process.

### 6.2. Gaussian Mixture Model

The probabilistic model that uses the expectation maximization algorithm is the GMM, and it is the best model that can be used for classification and prediction. It is a set of several Gaussians used to represent the clusters of data. In general, Gaussian density is defined as the following in a dimensional space:

(18) $$\begin{array}{c} p\left(X,\theta \right)=\overset{Q}{\underset{q=1}{\sum }}\alpha_{k}N\left(x;\mu_{q,\sum q}\right). \end{array}$$

A GMM is a type of probabilistic model that states that all generated data samples are derived from a mixture of finite Gaussian densities, which is a category of probabilistic models. As a result, the GMM models the allotment of a dataset by employing a number of Gaussian density estimates [61].

### 6.3. Detrended Fluctuation Analysis

The DFA has been used for a wide range of problems in a wide range of domains in biomedical engineering, including DNA sequences, heart rate variations, and human gait analysis, among others [62]. DFA is used to calculate a long range of power laws or scaling analysis for noisy time series data. DFA is a popular fractal methodology for detecting lengthy correlations in noisy nonstationary time series. Long-term correlations in noisy nonstationary time series are often detected using DFA. Long-range correlation is the slow decay of statistical reliance.

For the time series data or signal, *s*(*i*) for *I* = 1, 2, 3, 4, ⋯*p*.

where *p* is the maximum length of the data. To find the profile of the signal

(19) $$\begin{array}{c} m\left(q\right)=\overset{q}{\underset{i=1}{\sum }}\left[s\left(i\right)-\langle s\rangle \right]. \end{array}$$

After that, divide the signal profile *m* (*q*) into boxes of equal length. Afterwards, for each box, compute the trend of the signal in that box by fitting a polynomial of order “1” to the data (*q*). Detrend the signal is achieved by subtracting the trend from each of the signal boxes. When the detrended signal from the profile is integrated as *G* (*p*), the root mean square of the fluctuation is obtained.

(20) $$\begin{array}{c} G\left(p\right)=\sqrt{\frac{1}{P}\overset{P}{\underset{q=1}{\sum }}{\left[m\left(q\right)-m_{n}\left(q\right)\right]}^{2}}. \end{array}$$

### 6.4. Nonlinear Regression

When it comes to smoothing and classification, NR is a statistical method that can be used with both linear and nonlinear inputs. As an example of this, Nonlinear Regression is used to depict system functionality by using nonlinear variables as inputs to the model. As a result, the data collected will be fitted with a curve and categorized according to its classification. A Nonlinear Regression can be mathematically modelled as the classifier reaction is calculated by the values of the model equation [63].

It is expressed as,

(21) $$\begin{array}{c} Fn=x\left(c_{n},\theta \right)+S_{nn}, \end{array}$$

where the expectation function is denoted as *x*, and *c*_*n*_ denotes the vector if associated independent variable or regressor variables for the *n*^th^ case. One of the derivatives of the expectation function should depend on at least one of the parameters in nonlinear models. In order to distinguish between linear and nonlinear models, expectation function in a nonlinear model, is used as a parameter.

### 6.5. Bayesian Linear Discriminant Classifier

BLDC, which is a systematized and simple extension of Fisher's Linear Discriminant Classifier, aims to reduce the risk involved with the categorization choice as much as possible. It is capable of dealing with information with a high degree of complexity and noise. Since it depends on the Bayes decision rule, the error probability is reduced [64]. The major assumption in Bayesian regression is that the target *x* has a linear relation to the vector *k* with an additive white Gaussian noise *n*, it is expressed as,

(22) $$\begin{array}{c} x=q^{T}k+n, \end{array}$$

for the weight denoted as *q*. The likelihood function given as

(23) $$\begin{array}{c} p\left(\frac{D}{\beta ,q}\right)={\left(\frac{\beta }{2\pi }\right)}^{n/2}\exp\left(-\frac{\beta }{2}{\left\|K^{T}q-x\right\|}^{2}\right), \end{array}$$

where *x* represents a vector containing the regression targets, *K* denotes the matrix obtained from the horizontal stacking of the training feature vectors, *D* represents the pair {*K*, *x*}, *β* is the inverse variance of the noise, and *N* is the number of samples in the training set.

### 6.6. Linear Regression

Statistical methods such as linear regression have been around for a long time. As shown in this example, the output of the classifiers is defined by the following combination of the parameters used as inputs. It represents the most basic type of linear regression. A linear regression expressed as

(24) $$\begin{array}{c} Z=p+qY. \end{array}$$

*Y* represents the input and *Z* represents the output. In this equation, the slope of the line is *q*, and the intercept (the value of *z* when *y* =0) is *a*. Increased accuracy of classification can be achieved by employing a technique to determine the slope variable *p* [65]. An easy way to arrive at a slope vector matrix is to apply the minimum mean square error condition.

### 6.7. *K*-Nearest Neighbor

The *K*-Nearest Neighbor technique is a relatively basic procedure for classifying samples based on the majority voting among their neighbours and is performed as follows. Each sample is taken one at a time from the test set. Secondly, an estimate of the Euclidean distance between the test sample and all of the training set is made. And then, the class labels of the KNN training samples of the test labels are determined, where *K* is always an odd integer. Finally, each sample is given to a class that has the greatest number of training samples in the *K*-Nearest Neighbors clustering algorithm [66].

Given two different input vectors *x*_*n*_ and *x*_*m*_, their distance is given by

(25) $$\begin{array}{c} d_{n,n}=\sqrt{\overset{d}{\underset{i=1}{\sum }}{\left|X_{n,i}-X_{m,i}\right|}^{p}}. \end{array}$$

*X*_*n*_ and *X*_*m*_ are two separate input vectors and *d* is Euclidean distance.

## 7. Results and Discussions

For each sample used as input to the classifiers, 660 data points from FCM and 3300 data points from SDA, Hilbert, DCT, and FFT feature extraction techniques were used. Classifiers are designed to precisely divide a dataset into cancer cells and normal datasets, which is the primary objective of this algorithm. In order to assess the classification performance of classifiers, it is quite usual to employ the confusion matrix. The confusion matrix is a very simple idea; it is a square matrix that includes all the different classes, both horizontally and vertically. Mention the classes as the results obtained on the top of a table with the targets on the right.

Confusion matrix is derived from the four elements True Positive (TP), True Negative (TN), False Positive (FP), and False Negative (FN).

### 7.1. Classification without Feature Selection

After applying majority voting to the ensemble of classifiers, the output of the ensemble of classifiers is the computed class labels for the test samples. In order to compare the computed and targeted outputs, a confusion matrix was produced, and the resulting representation is displayed in Table 2. In order to assess how well the classifier performs based on these values, the accuracy, precision, and error rate have all been measured and reported for both normal and ovarian microarray gene data. The mean square error (MSE) of the classifiers is determined.

Table 3 shows the average values of MSE for FCM, SDA, Hilbert, FFT, and DCT features for GMM, DFA, NLR, BDLC, LR, and KNN classifiers. The table also gives the TP, TN, FP, and FN values for extracted features for GMM, DFA, NLR, BDLC, LR, and KNN classifiers. In the FCM feature, the LR classifier obtains the minimum MSE of 3.03e-05 and the NLR classifier attains the maximum MSE of 2.10e-04. In the SDA feature, the NLR classifier obtains the minimum MSE of 2.38E-06 and the LR classifier attains the maximum MSE of 2.34E-04. For the Hilbert transformed feature, the BDLC classifier obtains the minimum MSE of 1.80E-05 and the NLR classifier attains the maximum MSE of 2.10E-04. For the FFT feature, the GMM classifier obtains a minimum MSE of 2.77E-05 and the KNN classifier attains a maximum MSE of 1.34E-04. For the DCT feature, the LR classifier obtains a minimum MSE of 1.19E-05 and the KNN classifier attains a maximum MSE of 2.21E-04.

The features are extracted from the microarray gene data using FCM, SDA, Hilbert, DCT, and FCT methods for both normal and ovarian gene data. The extracted features are provided to the six classification models to analyze the performance. The performance measures of six classifiers are shown in Table 4. DFA classifiers attain the highest accuracy for FCM features among the other classifiers at 74%, with a high precision of 66.667%, a high F1 score of 78.689%, with an MCC of 0.535%, with high Jaccard metrics of 64.865%, and a CSI value of 62.667%. For FCM features among the other classifiers, DFA has a lower error rate of 26%. KNN provides lower parametric values, such as accuracy of 60%, MCC of 0.203, and CSI of 26.621%.

In SDA feature, compared with the other classifiers, NLR classifiers outperformed with the highest accuracy of 92%, with high precision of 88.889%, a high F1 score of 92.308%, with MCC of 0.843%, with high Jaccard metrics of 85.714%, and a CSI value of 84.889%. For SDA features, among the other classifiers, NLR has the lowest error rate at 8%. The NLR classifier error rate value is drastically reduced. KNN gives the lowest parametric values like accuracy of 55%, MCC of 0.100, and 10.902% as CSI. BDLC classifiers have the best accuracy of 77%, with precision of 78.723%, an F1 score of 76.289%, MCC of 0.541%, high Jaccard metrics of 61.667%, and a CSI value of 52.723% for Hilbert features. The other classifiers have lower accuracy. For Hilbert features, among the other classifiers, KNN has a low accuracy of 55% and a high error rate of 45%.

The error rate of the KNN classifier in SDA, Hilbert, and DCT features reaches as high as 45%. Among the other classifiers, GMM classifiers achieve the highest accuracy for FFT features at 75%, with precision of 80.448%, an F1 score of 72.527%, MCC of 0.508%, Jaccard metrics of 56.897%, and a CSI value of 46.448%. For FFT features, among the other classifiers, GMM has a low error rate of 25%. The LR classifier for FFT features has an accuracy rate of 58% and an error rate of 42%. DFA classifiers attain the highest accuracy for DCT features among the other classifiers at 82%, an F1 score of 83.333%, with MCC of 0.836%, with high Jaccard metrics of 71.429%, and a CSI value of 67.657%. For DCT features among the other classifiers, KNN has a low error rate of 45% and 55% accuracy.

The comparison graph of the accuracy for the six classifiers is shown in Figure 6. Without selecting the features, the NLR classifiers give the best accuracy and outperform other classifiers. For all the features, the accuracy, precision, and Jaccard metrics are high and the error rate is lower.

### 7.2. Classification with Feature Selection

The extracted features are given to the six classifiers to analyze the performance after the feature selection. The average MSE and confusion matrix for normal and ovarian data with correlation distance feature selection is shown in Table 5. The performance measures with feature selection of six classifiers are shown in Table 6. For all the features, the accuracy, precision, and Jaccard metrics are high and the error rate is lower. The comparison graph of the accuracy for the six classifiers is shown in Figure 7. Without selecting the features, the NLR classifiers give the best accuracy and outperform other classifiers.

Table 6 shows the average values of MSE for FCM, SDA, Hilbert, FFT, and DCT features for GMM, DFA, NLR, BDLC, LR, and KNN classifiers with feature selection. The table also gives the TP, TN, FP, and FN values for extracted features for GMM, DFA, NLR, BDLC, LR, and KNN classifiers with feature selection.

In the FCM feature, the LR classifier obtains a minimum MSE of 2.36E-05 and the KNN classifier attains a maximum MSE of 0.000125. In the SDA feature, the GMM classifier obtains a minimum MSE of 2.45E-05 and the NLR classifier attains a maximum MSE of 0.000262. For the Hilbert transformed feature, the BDLC classifier obtains a minimum MSE of 1.3E-05 while the LR classifier attains a maximum MSE of 0.000192. For the FFT feature, the DFA classifier obtains a minimum MSE of 6.42E-06 and the LR classifier attains a maximum MSE of 0.000187. For the DCT feature, the GMM classifier obtains a minimum MSE of 4.64E-06 and the DFA classifier attains a maximum MSE of 8.89E-05.

While the NLR classifier obtains 92% accuracy for SDA features when no features are selected, the KNN classifier only achieves 55% accuracy for SDA, Hilbert, and DCT features when no features are selected. The NLR classifier outperforms the other five classifiers in this situation. For FCM features, the LR classifier has the highest classification accuracy of 77% compared with other classifiers and also has the highest F1 score of 79.279, with a low error rate of 23. KNN classifiers have a low accuracy of 56% for FCM features with a high error rate of 44%. For SDA features, the GMM classifier has the highest classification accuracy of 76% compared with other classifiers and also has a high F1 score of 77.778, with a low error rate of 24. NLR classifiers have a low accuracy of 53% for SDA features with a high error rate of 47%. For Hilbert features, the BDLC classifier has a high classification accuracy of 82% compared with other classifiers and also has a high F1 score of 83.333, with a low error rate of 18. GMM classifiers have a low accuracy of 63% for Hilbert features with a high error rate of 37%. For FFT features, the DFA classifier has the highest classification accuracy of 86% compared with other classifiers and also has a high F1 score of 86.538, with a low error rate of 14. BDLC classifiers have a low accuracy of 56% for FFT features with a high error rate of 44%.

GMM outperforms among the other classifiers with the highest accuracy of 88%, with a high precision of 85.185%, an F1 score of 88.462%, with a high MCC of 0.762, with the lowest error rate of 12, and a CSI value of 77.185 for DCT features; NLR achieves the lowest accuracy of 53% for SDA features when the feature selection is done. The lowest accuracy of all of the classifiers tested.

Compared to other classification algorithms tested in this study, the result reveals that NLR delivers the best and highest classification accuracy for all of the data. As a result, the algorithm is more general than earlier classification algorithms. KNN, on the other hand, has the lowest accuracy of all the algorithms.

## 8. Conclusion

Ovarian cancer is the most common female malignancy. Computer-aided diagnosis is required to perform the proper diagnosis. Microarray technology allows for the simultaneous monitoring of thousands of genes under certain conditions. Microarray technology allows the study of gene expression and generates a lot of data. As a result of the curse of dimensionality and the tiny model space, further processing is difficult. In this research work, the 33000 microarray gene data for 100 samples are used, and with the help of ANOVA method, 16000 prominent genes were selected. The features are extracted using FCM, SDA, Hilbert, DCT, and FFT techniques, and the statistical parameters are analyzed. By correlation distance, the 45 genes are selected for classification. With and without feature selection by correlation distance for the extracted features, the datasets are classified by classifiers to get the best accuracy rate. The best results obtained by NLR classifiers were 92% accuracy for SDA features without feature selection. Mathematical-based feature selection has less accuracy compared to without feature selection. The future work will be the proposed feature selection techniques by various heuristic algorithms and to enhance the classification accuracy for the microarray gene data.

## Figures and Tables

**Figure 1:** Schematic representation of the methodology of the classification for ovarian and normal tissues from microarray gene data.

**Figure 2:** Volcano plot for ovarian and normal microarray gene data.

**Figure 3:** FCM feature histogram for normal and ovarian cancer microarray gene data.

**Figure 4:** Scatter plot of ovarian cancer and normal to FCM feature output.

**Figure 5:** Normal probability plot for ovarian cancer of SDA feature output.

**Figure 6:** Accuracy analyses without feature selection by correlation distance of classifiers.

**Figure 7:** Accuracy analyses with feature selection by correlation distance of classifiers.

**Table 1:** Statistical parameters of clustering- and transform-based feature extraction for ovarian and normal data.

Statistical parameters	FCM		SDA		Hilbert		FFT		DCT	
	Ovarian	Normal	Ovarian	Normal	Ovarian	Normal	Ovarian	Normal	Ovarian	Normal
Mean	0.60958	0.61855	12.09748	0.21740	0.49855	0.49357	0.00810	0.00734	0.00731	0.00663
Std dev	0.0722	0.06839	7.56472	0.15279	0.09348	0.08900	0.01736	0.01736	0.01741	0.01740
Variance	0.0052	0.00470	1.14519	0.02336	0.00875	0.00794	0.00030	0.00030	0.00030	0.00030
Skewness	1.8415	1.98612	75.87783	1.69340	1.39834	1.62165	56.62020	56.73028	56.23927	56.42410
Kurtosis	4.4688	5.03687	122.1244	2.92235	2.89985	3.65340	3236.49200	3244.93585	3207.17014	3221.32183
Pearson	0.9653	0.94569	46.05714	0.91892	0.94541	0.91843	0.99891	0.99861	0.99807	0.99757
*T*-test	0.0214	0.01497	1.0306	0.00714	0.00389	0.00184	0.00341	0.00005	0.01034	0.00226
Sample entropy	9.3663	9.36632	582.756	11.638	11.688	11.68825	10.68857	10.68849	11.68772	11.68772

**Table 2:** Performance metrics of the classifiers.

Performance metrics	Description of metrics	Derived from confusion matrix
Accuracy	Average of no of samples identified as positive to no. of samples identified as negative	$Ac=\frac{\left(TN+TP\right)}{\left(TN+FN+TP+FP\right)}$
Precision	From all correct predictions, accurately predicted.	$PR=\frac{TP}{\left(TP+FP\right)}$
MSE	Average of the squared error	$MSE=\frac{1}{N}\overset{N}{\underset{i=1}{\sum }}{\left(y_{i}-y_{i}^{\wedge }\right)}^{2}$
F1 score	Mean of precision and recall to get classification accuracy for a specific class	$F1=\frac{2*TP}{\left(2*TP+FP+FN\right)}$
Mathews correlation coefficient	Pearson correlation between true and attained output	$MCC\frac{\left(TP*TN-FP*FN\right)}{\sqrt{\left(\left(TP+FP\right)*\left(TN+FP\right)*\left(TN+FN\right)\right)}}$
Fowlkes mallows index	Measure of similarity between clustering	$FM=\sqrt{\frac{TP}{TP+FP}.\frac{TP}{TP+FN}}$
Error rate	Based on the number of observations, the sum of all inaccurate predictions.	$ErR=\frac{\left(FP+FN\right)}{\left(TP+FN+TN+FP\right)}$
Jaccard metric	The predicted real positives outnumbered the actual positives, whether they happened to be real or predicted.	$Jac=\frac{TP}{\left(TP+FP+FN\right)}$
Classification success index	Averaging the class-specific symmetric measure of overall class	*CSI* = *PPV* + *SEN* − 100

**Table 3:** Average MSE and confusion matrix for normal and ovarian data without feature selection.

Feature extraction	Classifiers	TP	TN	FP	FN	MSE
FCM	GMM	44	26	24	6	1.82e-04
	Detrend FA	48	26	24	2	2.00e-04
	NLR	47	26	24	3	2.10e-04
	BDLC	39	27	23	11	1.06e-04
	LR	40	27	23	10	3.03e-05
	KNN	34	26	24	16	1.82e-04

SDA	GMM	42	43	7	8	4.62E-06
	Detrend FA	46	40	10	4	6.98E-06
	NLR	48	44	6	2	2.38E-06
	BDLC	35	26	24	15	2.06E-04
	LR	36	26	24	14	2.34E-04
	KNN	28	27	23	22	1.75E-04

Hilbert Transform	GMM	30	27	23	20	1.85E-04
	Detrend FA	47	26	24	3	2.01E-04
	NLR	48	26	24	2	2.10E-04
	BDLC	37	40	10	13	1.80E-05
	LR	33	42	8	17	2.67E-05
	KNN	28	27	23	22	1.68E-04

FFT	GMM	33	42	8	17	2.77E-05
	Detrend FA	45	28	22	5	7.31E-05
	NLR	45	29	21	5	4.33E-05
	BDLC	34	34	16	16	3.97E-05
	LR	29	29	21	21	7.87E-05
	KNN	26	41	9	24	1.34E-04

DCT	GMM	36	41	9	14	1.73E-05
	Detrend FA	45	37	13	5	1.19E-05
	NLR	46	29	21	4	3.59E-05
	BDLC	37	36	14	13	2.68E-05
	LR	31	29	21	19	6.92E-05
	KNN	29	26	24	21	2.21E-04

**Table 4:** Performance measures of classifiers for normal and ovarian data without feature selection.

Feature extraction	Classifiers	Performance measures							
		Accuracy	Precision	F1Score	MCC	FM	Error rate	Jaccard metric	CSI
FCM	GMM	70	64.706	74.576	0.429	0.755	30	59.459	52.706
	Detrend FA	74	66.667	78.689	0.535	0.800	26	64.865	62.667
	NLR	73	66.197	77.686	0.507	0.789	27	63.514	60.197
	BDLC	66	62.903	69.643	0.330	0.700	34	53.425	40.903
	LR	67	63.492	70.796	0.352	0.713	33	54.795	43.492
	KNN	60	58.621	62.963	0.203	0.631	40	45.946	26.621

SDA	GMM	85	85.714	84.848	0.700	0.849	15	73.684	69.714
	Detrend FA	86	82.143	86.792	0.725	0.869	14	76.667	74.143
	NLR	92	88.889	92.308	0.843	0.924	8	85.714	84.889
	BDLC	61	59.322	64.220	0.224	0.644	39	47.297	29.322
	LR	62	60.000	65.455	0.245	0.657	38	48.649	32.000
	KNN	55	54.902	55.446	0.100	0.554	45	38.356	10.902

Hilbert Transform	GMM	57	56.604	58.252	0.140	0.583	43	41.096	16.604
	Detrend FA	73	66.197	77.686	0.507	0.789	27	63.514	60.197
	NLR	74	66.667	78.689	0.535	0.800	26	64.865	62.667
	BDLC	77	78.723	76.289	0.541	0.763	23	61.667	52.723
	LR	75	80.488	72.527	0.508	0.729	25	56.897	46.488
	KNN	55	54.902	55.446	0.100	0.554	45	38.356	10.902

FFT	GMM	75	80.488	72.527	0.508	0.729	25	56.897	46.488
	Detrend FA	73	67.164	76.923	0.489	0.777	27	62.500	57.164
	NLR	74	68.182	77.586	0.507	0.783	26	63.380	58.182
	BDLC	68	68.000	68.000	0.360	0.680	32	51.515	36.000
	LR	58	58.000	58.000	0.160	0.580	42	40.845	16.000
	KNN	67	74.286	61.176	0.356	0.622	33	44.068	26.286

DCT	GMM	77	80.000	75.789	0.543	0.759	23	61.017	52.000
	Detrend FA	82	77.586	83.333	0.648	0.836	18	71.429	67.586
	NLR	75	68.657	78.632	0.532	0.795	25	64.789	60.657
	BDLC	73	72.549	73.267	0.460	0.733	27	57.813	46.549
	LR	60	59.615	60.784	0.200	0.608	40	43.662	21.615
	KNN	55	54.717	56.311	0.100	0.563	45	39.189	12.717

**Table 5:** Average MSE and confusion matrix for normal and ovarian data with correlation distance feature selection.

Feature extraction	Classifiers	TP	TN	FP	FN	MSE
FCM	GMM	30	36	14	20	4.58E-05
	Detrend FA	28	41	9	22	5.41E-05
	NLR	30	33	17	20	5.54E-05
	BDLC	36	29	21	14	4.82E-05
	LR	44	33	17	6	2.36E-05
	KNN	29	27	23	21	0.000125

SDA	GMM	42	34	16	8	2.45E-05
	Detrend FA	41	27	23	9	9.06E-05
	NLR	26	27	23	24	0.000262
	BDLC	43	29	21	7	4.18E-05
	LR	34	29	21	16	5.55E-05
	KNN	28	27	23	22	0.000142

Hilbert Transform	GMM	29	34	16	21	5.53E-05
	Detrend FA	49	27	23	1	0.000105
	NLR	44	35	15	6	1.71E-05
	BDLC	45	37	13	5	1.3E-05
	LR	44	26	24	6	0.000192
	KNN	33	37	13	17	3.43E-05

FFT	GMM	29	42	8	21	4.53E-05
	Detrend FA	45	41	9	5	6.42E-06
	NLR	35	27	23	15	9.02E-05
	BDLC	29	27	23	21	0.000163
	LR	35	26	24	15	0.000187
	KNN	27	31	19	23	0.000115

DCT	GMM	46	42	8	4	4.64E-06
	Detrend FA	46	27	23	4	8.89E-05
	NLR	45	28	22	5	7.92E-05
	BDLC	37	36	14	13	2.28E-05
	LR	34	42	8	16	2.42E-05
	KNN	28	33	17	22	6.8E-05

**Table 6:** Performance measures of classifiers for ovarian data with feature selection.

Feature extraction	Classifiers	Performance measures							
		Accuracy	Precision	F1 score	MCC	FM	Error rate	Jaccard metric	CSI
FCM	GMM	66	68.182	63.830	0.322	0.640	34	46.875	28.182
	Detrend FA	69	75.676	64.368	0.394	0.651	31	47.458	31.676
	NLR	63	63.830	61.856	0.260	0.619	37	44.776	23.830
	BDLC	65	63.158	67.290	0.303	0.674	35	50.704	35.158
	LR	77	72.131	79.279	0.554	0.797	23	65.672	60.131
	KNN	56	55.769	56.863	0.120	0.569	44	39.726	13.769

SDA	GMM	76	72.414	77.778	0.527	0.780	24	63.636	56.414
	Detrend FA	68	64.063	71.930	0.375	0.725	32	56.164	46.063
	NLR	53	53.061	52.525	0.060	0.525	47	35.616	5.061
	BDLC	72	67.188	75.439	0.458	0.760	28	60.563	53.188
	LR	63	61.818	64.762	0.261	0.648	37	47.887	29.818
	KNN	55	54.902	55.446	0.100	0.554	45	38.356	10.902

Hilbert Transform	GMM	63	64.444	61.053	0.261	0.611	37	43.939	22.444
	Detrend FA	76	68.056	80.328	0.579	0.817	24	67.123	66.056
	NLR	79	74.576	80.734	0.590	0.810	21	67.692	62.576
	BDLC	82	77.586	83.333	0.648	0.836	18	71.429	67.586
	LR	70	64.706	74.576	0.429	0.755	30	59.459	52.706
	KNN	70	71.739	68.750	0.401	0.688	30	52.381	37.739

FFT	GMM	71	78.378	66.667	0.435	0.674	29	50.000	36.378
	Detrend FA	86	83.333	86.538	0.722	0.866	14	76.271	73.333
	NLR	62	60.345	64.815	0.243	0.650	38	47.945	30.345
	BDLC	56	55.769	56.863	0.120	0.569	44	39.726	13.769
	LR	61	59.322	64.220	0.224	0.644	39	47.297	29.322
	KNN	58	58.696	56.250	0.161	0.563	42	39.130	12.696

DCT	GMM	88	85.185	88.462	0.762	0.885	12	79.310	77.185
	Detrend FA	73	66.667	77.311	0.497	0.783	27	63.014	58.667
	NLR	73	67.164	76.923	0.489	0.777	27	62.500	57.164
	BDLC	73	72.549	73.267	0.460	0.733	27	57.813	46.549
	LR	76	80.952	73.913	0.527	0.742	24	58.621	48.952
	KNN	61	62.222	58.947	0.221	0.590	39	41.791	18.222

## Data Availability

The microarray ovarian cancer database is accessible in ovarian cancer sample microarray gene data E-GEOD–69207, which was collected by the European Bioinformatics Institute (EMBL-EBI) and is openly accessible.
